The article "Significance of Laboratory Findings and Esophageal Varices in Male Patients With Decompensated Alcoholic Liver Cirrhosis: A Single-Center Experience" was published in 2025. Journal: Cureus.

# Significance of Laboratory Findings and Esophageal Varices in Male Patients With Decompensated Alcoholic Liver Cirrhosis: A Single-Center Experience

**DOI:** 10.7759/cureus.78274

**Published:** 2025-01-31

**Authors:** Goran Bokan, Marijana Kovacevic, Natasa Zdravkovic, Dejan Bokonjic, Maksim Kovacevic, Verica Prodanovic, Zoran Mavija

**Affiliations:** 1 Gastroenterology and Hepatology, University Clinical Centre of the Republika Srpska, Banja Luka, BIH; 2 Nephrology, Foca University Hospital, Foca, BIH; 3 Gastroenterology and Hepatology, University Clinical Center of Kragujevac, Kragujevac, SRB; 4 Pediatrics and Neonatology, Foca University Hospital, Foca, BIH; 5 Surgery, Foca University Hospital, Foca, BIH; 6 Cardiology, Foca University Hospital, Foca, BIH; 7 Gastroenterology, University Clinical Centre of the Republika Srpska, Banja Luka, BIH

**Keywords:** alcoholic liver cirrhosis, complications, decompensation, esophagus varices, laboratory parameters, male patients

## Abstract

Introduction

Alcoholic liver disease represents a growing global pandemic, particularly among younger men, and is one of the leading causes of premature death worldwide. Observing complications during the decompensation stage and monitoring disease progression dynamics using scoring systems are particularly important.

Materials and methods

This retrospective-prospective, descriptive, and analytical study included 123 male patients with a confirmed diagnosis of alcoholic liver cirrhosis, hospitalized at the Internal Medicine Clinic, University Clinical Centre of the Republic of Srpska in Banja Luka, Department of Gastroenterology and Hepatology. The study period spanned from January 2023 to January 2025, with the note that patient selection and monitoring began much earlier, in June 2021. After hospitalization, patients were followed monthly through a program of outpatient control examinations, with disease outcomes recorded. The study included all male patients over 18 years of age with a confirmed diagnosis of alcoholic liver cirrhosis and signed informed consent. Female patients and those with cirrhosis or other etiologies were excluded. For statistical data analysis, the Statistical Package for the Social Sciences (SPSS) version 29 (IBM Corp., Armonk, NY, USA) was used. The statistical analyses performed included median, standard deviation, analysis of variance, Student's t-test, chi-square test, and survival analysis.

Results

The mean age of the patients was 59.09±9.316 years. Most of them had anemia: 113 patients (91.86%) with decreased erythrocytes and 109 patients (88.62%) with decreased hemoglobin. Thrombocytopenia was observed in 104 patients (84.55%), while an increased mean corpuscular volume (MCV) was recorded in 68 patients (55.28%). Among biochemical parameters, the most common findings were increased bilirubin in 98 patients (79.67%), aspartate aminotransferase (AST) in 111 patients (90.24%), gamma-glutamyl transferase (GGT) in 109 patients (88.61%), and D-dimer in 110 patients (89.44%), while albumin levels were decreased in 107 patients (87.00%). Hyponatremia (decreased sodium) was observed in 63 patients (51.21%), and hypercalcemia (increased calcium) in 116 patients (94.30%). Jaundice was the most common external sign, present in 98 patients (79.67%), while ascites were noted in 86 patients (69.91%). Death during the first decompensation occurred in 31 patients (25.20%), of whom 17 (54.83%) died in the hospital. The leading cause of mortality is bleeding from esophageal varices.

The article "Significance of Laboratory Findings and Esophageal Varices in Male Patients With Decompensated Alcoholic Liver Cirrhosis: A Single-Center Experience" was published in 2025. Journal: Cureus.

Conclusion

Although a healthy liver performs over 200 distinct functions in the human body, a cirrhotic liver leads, one might say, to an even greater number of dysfunctions. This pathology is extremely complex, characterized by numerous complications and high treatment costs, which, despite all applied measures, do not ensure a favorable long-term prognosis without liver transplantation.

## Introduction

Alcohol is one of the most widely used psychoactive substances worldwide, deeply embedded in social and cultural contexts. While moderate alcohol consumption is often an integral part of social gatherings and traditions, excessive and prolonged intake can lead to severe health consequences, particularly affecting the liver. Alcoholic liver disease encompasses a spectrum of pathological changes caused by chronic alcohol consumption, ranging from fatty liver (steatosis) and alcoholic steatohepatitis to fibrosis, cirrhosis, and, in advanced stages, hepatocellular carcinoma [1-4].

Effective management of alcoholic liver disease requires a multidisciplinary approach, with absolute alcohol abstinence being the cornerstone of therapy. This is essential for slowing disease progression, reducing complications, and improving overall survival. In addition, treatment protocols include intensive nutritional support, targeted pharmacological and endoscopic interventions for managing complications, and an assessment of liver transplantation eligibility in advanced disease stages [5-8].

The primary objective of this study is to evaluate the significance of laboratory findings and the presence of esophageal varices in male patients with decompensated alcoholic liver cirrhosis and their association with mortality outcomes. A clear understanding of these factors may improve risk stratification and clinical management strategies for this patient population.

The article "Significance of Laboratory Findings and Esophageal Varices in Male Patients With Decompensated Alcoholic Liver Cirrhosis: A Single-Center Experience" was published in 2025. Journal: Cureus.

## Materials and methods

This retrospective-prospective, descriptive, and analytical study included 123 male patients with a confirmed diagnosis of alcoholic liver cirrhosis who were hospitalized at the Internal Medicine Clinic, University Clinical Centre of the Republic of Srpska in Banja Luka, Department of Gastroenterology and Hepatology. The study period spanned from January 2023 to January 2025, with patient selection and initial monitoring beginning in June 2021. Patients were followed monthly after hospitalization through an outpatient control program, with disease outcomes recorded.

Patient selection and inclusion criteria

Eligible participants were male patients over 18 years of age with a confirmed diagnosis of alcoholic liver cirrhosis based on clinical, biochemical, and imaging findings. Exclusion criteria included female patients, individuals with non-alcoholic liver cirrhosis (e.g., viral, autoimmune, or metabolic liver disease), and those with significant extrahepatic malignancies. Additionally, patients with severe chronic comorbidities that could significantly influence survival (e.g., advanced cardiovascular or pulmonary disease) were excluded. Only patients who provided signed informed consent were included in the study.

Data collection and diagnostic procedures

All necessary diagnostic work-up, including laboratory, microbiological, serological, radiological, and endoscopic evaluations, were conducted during the first hospitalization. Blood samples for hematological parameters (complete and differential blood count) were analyzed using the Sysmex XP 1000 device in the Central Laboratory. Biochemical parameters were assessed using the Abbott Alinity system, and coagulation parameters were measured with the Siemens BCS device.

Key laboratory values analyzed included erythrocytes, leukocytes, hemoglobin, mean corpuscular volume (MCV), platelets, glucose, bilirubin, liver enzymes (aspartate aminotransferase (AST), alanine aminotransferase (ALT), gamma-glutamyl transferase (GGT), lactate dehydrogenase (LDH), alkaline phosphatase (ALP)), urea, creatinine, ammonia, electrolytes (potassium (K+), sodium (Na+), chloride (Cl−), calcium (Ca2+)), phosphates, international normalized ratio (INR), albumin, total protein, C-reactive protein (CRP), and D-dimer.

Assessment of esophageal varices and cirrhosis decompensation

Esophageal varices were diagnosed via upper gastrointestinal endoscopy performed during hospitalization. The presence, size, and signs of recent bleeding (e.g., red wale signs) were documented. The primary causes of hospitalization in patients with decompensated cirrhosis were analyzed, with a particular focus on the significance of esophageal varices in mortality outcomes. Other complications of decompensated cirrhosis, including ascites, hepatic encephalopathy, spontaneous bacterial peritonitis, and hepatorenal syndrome, were also systematically recorded.

The article "Significance of Laboratory Findings and Esophageal Varices in Male Patients With Decompensated Alcoholic Liver Cirrhosis: A Single-Center Experience" was published in 2025. Journal: Cureus.

Statistical analysis

The statistical analysis of the obtained data was performed using the Statistical Package for the Social Sciences (SPSS), version 29 (IBM Corp., Armonk, NY, USA). The research results are presented as mean and standard deviation for variables with a normal distribution and as median with interquartile range for variables that do not follow a normal distribution. The statistical significance of differences in mean values between the examined groups will be determined using analysis of variance (ANOVA) and t-test for variables with a normal distribution, as well as the chi-square test for categorical variables.

## Results

The mean age of the subjects was 59.09±9.316. The oldest patient included in the study was 85 years old, while the youngest was 33 years old. The majority of patients, 113 of them (91.86%), had reduced erythrocyte values (below 4.5 x10⁹/L), the lowest being 1.78, while normal values were present in 6.5% of patients. Elevated values of leukocytes above 8 x10⁹/L were recorded in 34.95%, and normal values in 55.28%. Hemoglobin was lowered in 88.62% of patients, with the lowest value of 65, while normal values were present in only 11.38%. Elevated MCV values above 96 fL were present in 55.28%, while decreased MCV values below 80 fL were present in 6.5% of patients. Reduced values of platelets (below 150 x10⁹/L) were recorded in 84.55% of subjects, while 13% of patients had normal values. The highest recorded value of platelets was 477 x10⁹/L, while the minimum was 12 x10⁹/L (Table 1).

**Table 1:** Review of hemograms in hospitalized patients Statistical analysis was performed using the chi-square test.

Parameter	Category	Reference values	N	%	Min.	Max.	P-values
Red blood cells	Elevated	>5.3 x 10^12^/L	2	1.62	1.78	5.33	p<0.05
	Normal	4.5-5.3 x 10^12^/L	8	6.50			
	Decreased	<4.5 x 10^12^/L	113	91.86			
White blood cells	Elevated	>8 x 10^9^/L	43	34.95	2.03	27.10	p<0.05
	Normal	3-8 x 10^9^/L	68	55.28			
	Decreased	<3 x 10^9^/L	12	9.75			
Hemoglobin	Elevated	>181 g/L	0	0	65	159	p<0.05
	Normal	140-180 g/L	14	11.38			
	Decreased	>139 g/L	109	88.62			
Mean corpuscular volume	Elevated	>96 f/L	68	55.28	63.50	116.50	p<0.05
	Normal	80-96 f/L	47	38.21			
	Decreased	<80 f/L	8	6.5			
Plates	Elevated	>400 x 10^9^/L	3	2.43	12	477	p<0.05
	Normal	150-400 x 10^9^/L	16	13.00			
	Decreased	<150 x 10^9^/L	104	84.55			

The majority of patients, 98 (79.67%), had elevated total bilirubin values above 21.0 μmol/L, with a maximum value of 681 μmol/L, while 24 patients (19.51%) had values within the normal range from 5.0 to 21.0 μmol/L. Direct bilirubin was elevated in 117 patients (95.12%), with a maximum value of 654 μmol/L, while only six patients (4.87%) had values within the reference range of 0.0 to 3.4 μmol/L. AST activity was elevated in 111 patients (90.24%), with a maximum value of 2116 U/L, while 12 patients (9.75%) had values within the normal range of 0 to 35 U/L. Elevated ALT values were present in 46 patients (37.39%), with a maximum value of 1898 U/L, while most patients, 77 of them (62.60%), had values within the reference range. GGT activity was elevated in 109 patients (88.61%), with a maximum value of 1495 U/L, while 14 patients (11.38%) had normal values ranging from 0 to 35 U/L. LDH was elevated above 250 U/L in 41 patients (33.33%), with a maximum value of 5851 U/L, while normal LDH activity was recorded in 82 patients (66.67%). ALP activity was elevated in 63 patients (51.21%), with a maximum value of 1492 U/L, while in 58 patients (47.15%) it was within the normal range of 30 to 120 U/L, and only two patients (1.62%) had decreased values below 30 U/L. Elevated ammonia values above 60 μmol/L were recorded in 67 patients (54.47%), with a maximum value of 215 μmol/L, while in 56 patients (45.52%) ammonia was within the normal range of 16 to 60 μmol/L.

The article "Significance of Laboratory Findings and Esophageal Varices in Male Patients With Decompensated Alcoholic Liver Cirrhosis: A Single-Center Experience" was published in 2025. Journal: Cureus.

Total proteins in 71 patients (57.72%) were lowered below 66 g/L, while in 47 patients (38.21%) a normal concentration was recorded in the range from 66 to 83 g/L, and five patients (4.06%) had elevated values above 83 g/L. Albumin in 107 patients (87.00%) was lowered below 35 g/L, while in 16 patients (13.00%) it was within the normal range of 35 to 52 g/L.

CRP was elevated in 106 patients (86.17%), with a maximum value of 229 mg/L, while in 17 patients (13.82%) it was within the reference range. Glucose was elevated above 5.8 mmol/L in 56 patients (45.52%), while in 61 patients (49.59%) it was within the normal range of 3.9 to 5.8 mmol/L. Fourteen patients (11.38%) had elevated INR values above 2.0, while in 92 patients (74.79%), the value was within the normal range of 1.1 to 2.0. D-dimer was elevated in 110 patients (89.44%), with a maximum value of 11.4 µg/mL, while in 13 patients (10.56%) it was within the normal range below 0.5 µg/mL (Table 2).

**Table 2:** Review of hepatogram and liver synthetic function in hospitalized patients Statistical analysis was performed using the chi-square test.

Parameter	Category	Reference values	N	%	Min.	Max.	P-values
Total bilirubin	Elevated	>21.0 U/L	98	79.67	3.40	681	p<0.05
	Normal	5.0-21.0 U/L	24	19.51			
	Decreased	<5.0 U/L	1	0.81			
Conjugated bilirubin	Elevated	>3.4 U/L	117	95.12	0.2	654	p<0.05
	Normal	0.0-3.4 U/L	6	4.87			
Aspartate aminotransferase	Elevated	>35.0 U/L	111	90.24	7.30	2116	p<0.05
	Normal	0-35.0 U/L	12	9.75			
Alanine aminotransferase	Elevated	>35.0 U/L	46	37.39	1	1898	p<0.05
	Normal	0-35.0 U/L	77	62.60			
Gamma-glutamyl transferase	Elevated	>35.0 U/L	109	88.61	4.74	1495	p<0.05
	Normal	0-35.0 U/L	14	11.38			
Lactate dehydrogenase	Elevated	>250 U/L	41	33.33	85	5851	p<0.05
	Normal	0-250 U/L	82	66.67			
Alkaline phosphatase	Elevated	>120 U/L	63	51.21	1.30	1492	p<0.05
	Normal	30-120 U/L	58	47.15			
	Decreased	<30 U/L	2	1.62			
Ammonia	Elevated	>60 umol/L	67	54.47	26	215	p<0.05
	Normal	16-60 umol/L	56	45.52			
	Decreased	<16 umol/L	0	0			
Total protein	Elevated	>83 g/L	5	4.06	32.30	88.80	p<0.05
	Normal	66-83 g/L	47	38.21			
	Decreased	<66 g/L	71	57.72			
	Elevated	>52 g/L	0	0	16	48	p<0.05
Albumin	Normal	35-52 g/L	16	13.00			
	Decreased	<35 g/L	107	87.00			
	Elevated	>5.0 g/L	106	86.17	0.50	229	p<0.05
C-reactive protein	Elevated	>5.0 mg/L	106	86.17	0.50	229	p<0.05
	Normal	0.0-5.0 mg/L	17	13.82			
Glucose	Elevated	>5.8 mmol/L	56	45.52	3.2	28	p<0.05
	Normal	3.9-5.8 mmol/L	61	49.59			
	Decreased	<3.9 mmol/L	6	4.87			
International normalized ratio	Elevated	>2.0	14	11.38	0.94	5.20	p<0.05
	Normal	1.1- 2.0	92	74.79			
	Decreased	<1.1	17	13.82			
D-dimer	Elevated	>0.5µg/mL	110	89.44	0.69	11.4	p<0.05
	Normal	<0.5 µg/mL	13	10.56			

The analysis of laboratory parameters related to renal function and electrolytes in hospitalized patients with alcoholic cirrhosis is presented in Table 3. Urea was elevated above 7.2 mmol/L in 65 patients (52.84%), with a maximum value of 55.20 mmol/L. In 55 patients (44.71%), urea levels were within the normal range of 2.8 to 7.2 mmol/L, while in three patients (2.43%), levels were decreased below 2.8 mmol/L, with a minimum recorded value of 1.50 mmol/L. Creatinine was elevated above 84 µmol/L in 70 patients (56.91%), with a maximum value of 702 µmol/L. In 52 patients (42.27%), creatinine was within normal limits (45 to 84 µmol/L), and in one patient (0.81%), creatinine was below the normal range, with a value of less than 45 µmol/L. Potassium K⁺) was elevated above 5.1 mmol/L in four patients (3.25%), with a maximum value of 6.60 mmol/L. In 98 patients (79.64%), potassium levels were within the normal range of 3.5 to 5.1 mmol/L, and in 21 patients (17.07%), potassium was reduced below 3.5 mmol/L, with a minimum value of 2.19 mmol/L. Sodium (Na⁺) was elevated above 146 mmol/L in one patient (0.81%), while in 59 patients (47.96%), sodium was within the normal range of 136 to 146 mmol/L. In 63 patients (51.21%), sodium was decreased below 136 mmol/L, with a minimum value of 110 mmol/L. Calcium (Ca²⁺) was elevated above 1.29 mmol/L in 116 patients (94.30%), with a maximum value of 2.75 mmol/L. Only four patients (3.25%) had calcium levels within the normal range of 1.15 to 1.29 mmol/L, and in three patients (2.43%), calcium was decreased below 1.15 mmol/L, with a minimum value of 1.07 mmol/L. Chlorides (Cl⁻) were elevated above 106 mmol/L in 25 patients (20.32%), with a maximum value of 145 mmol/L. In 70 patients (56.91%), chloride concentrations were within normal limits (98 to 106 mmol/L), and in 28 patients (22.76%), chloride levels were decreased below 98 mmol/L, with a minimum value of 59 mmol/L. Phosphates (P) were elevated above 1.45 mmol/L in 13 patients (10.56%), with a maximum value of 3.21 mmol/L. In 73 patients (59.34%), phosphate levels were within the normal range (0.87 to 1.45 mmol/L), and in 37 patients (30.08%), phosphates were reduced below 0.87 mmol/L, with a minimum value of 0.31 mmol/L.

The article "Significance of Laboratory Findings and Esophageal Varices in Male Patients With Decompensated Alcoholic Liver Cirrhosis: A Single-Center Experience" was published in 2025. Journal: Cureus.

**Table 3:** Review of nitrogenous substances and ionograms in hospitalized patients Statistical analysis was performed using the chi-square test.

Parameter	Category	Reference values	N	%	Min.	Max.	P-values
Urea	Elevated	>7.2 mmol/L	65	52.84	1.50	55.20	p<0.05
	Normal	2.8-7.2 mmol/L	55	44.71			
	Decreased	<2.8 mmol/L	3	2.43			
Creatinine	Elevated	>84 umol/L	70	56.91	7	702	p<0.05
	Normal	45-84 umol/L	52	42.27			
	Decreased	<45 umol/L	1	0.81			
Potassium	Elevated	>5.1 mmol/L	4	3.25	2.19	6.60	p<0.05
	Normal	3.5-5.1 mmol/L	98	79.64			
	Decreased	<3.5 mmol/L	21	17.07			
Sodium	Elevated	>146 mmol/L	1	0.81	110	148	p<0.05
	Normal	136-146 mmol/L	59	47.96			
	Decreased	<136 mmol/L	63	51.21			
Calcium	Elevated	>1.29 mmol/L	116	94.30	1.07	2.75	p<0.05
	Normal	1.15-1.29 mmol/L	4	3.25			
	Decreased	<1.15 mmol/L	3	2.43			
Chlorides	Elevated	>106 mmol/L	25	20.32	59	145	p<0.05
	Normal	98-106 mmol/L	70	56.91			
	Decreased	<98 mmol/L	28	22.76			
Phosphate	Elevated	>1.45	13	10.56	0.31	3.21	p<0.05
	Normal	0.87-1.45 mmol/L	73	59.34			
	Decreased	<0.87	37	30.08			

Ascites is the most common complication, registered in 86 patients, which makes up 69.91% of the sample. Variceal hemorrhage was identified in 25 patients or 20.32% of the sample. Jaundice, although more common among external manifestations, was recorded as a clinically significant complication in seven patients, representing 5.69% of the total. Hepatic encephalopathy was registered in 15 patients or 12.19% of the sample. The dominant complications in the first decompensation of alcoholic liver cirrhosis are presented in Figure 1. Statistical analysis determined that p<0.05, which means that there is a statistically significant difference in the distribution of complications of liver cirrhosis, with a predominance of ascites.

The article "Significance of Laboratory Findings and Esophageal Varices in Male Patients With Decompensated Alcoholic Liver Cirrhosis: A Single-Center Experience" was published in 2025. Journal: Cureus.

**Figure 1:** Dominant complication in the first decompensation

Table 4 and Table 5 present the frequency of esophageal varicose and variceal bleeding in the subjects by grade. Grade I was observed in 27 patients (34.17%), of whom three patients (11.11%) experienced variceal bleeding. Grade II was registered in 30 patients (37.97%), of which 12 patients (40%) had variceal bleeding. Grade III varices were registered in 18 patients (22.78%), of whom nine patients (50%) had variceal bleeding. Grade IV varicices were registered in four patients (5.06%), of which one patient (25%) had variceal bleeding.

**Table 4:** Number of esophageal varices in hospitalized patients

Esophageal varices	N	%
Present	79	64.23%
Absent	44	35.77%
Total	123	

**Table 5:** Overview of the frequency of varices and bleeding varices in liver cirrhosis

Grade (Paquet classification)	N per grade	%	N of bleeding varices	%
I	27	34.17	3	11.11%
II	30	37.97	12	40%
III	18	22.78	9	50%
IV	4	5.06	1	25%
Total	79	Total	25	

Grades II and III esophageal varices pose the highest risk of bleeding, while smaller Grade I varices have a lower rate of complications. There is a statistically significant difference in the frequency of variceal bleeding among patients with different grades of varices (p<0.05).

Mortality due to variceal bleeding was observed in 14/123 (11.38%) patients during hospitalization, while in four patients it was registered during outpatient follow-up (Table 6). A p-value of less than 0.05 indicates a statistically significant association between the degree of variceal bleeding and mortality.

**Table 6:** Mortality in relation to the degree of varicosity

Degree of varicosity	N	% of total
I	0	0
II	6	42.85%
III	7	50%
IV	1	7.15%
Total	14	

## Discussion

Alcoholism, global alcohol consumption, and alcoholic liver disease represent complex public health challenges, with serious consequences for individuals and society as a whole. Alcoholism, also known as alcohol addiction, is a widespread problem worldwide. People struggling with alcoholism often face difficulties controlling their alcohol consumption, leading to numerous health, social, and economic problems. Factors contributing to the development of alcoholism include genetic predisposition, stress, trauma, social pressures, and the easy availability of alcohol [1-3].

Alcoholic liver cirrhosis is the terminal stage of alcoholic liver disease, characterized by permanent liver damage where healthy tissue is replaced by scarring and fibrosis. This process disrupts normal liver function, causing serious complications, including liver failure, portal hypertension, ascites, esophageal varices, encephalopathy, and hepatocellular carcinoma. Liver cirrhosis is the most common indication for liver transplantation, and without timely medical intervention, it can be fatal.

The article "Significance of Laboratory Findings and Esophageal Varices in Male Patients With Decompensated Alcoholic Liver Cirrhosis: A Single-Center Experience" was published in 2025. Journal: Cureus.

The pathogenesis of alcoholic cirrhosis begins with prolonged and excessive alcohol consumption, causing inflammation and damage to hepatocytes. Alcohol is metabolized in the liver by enzymes such as alcohol dehydrogenase (ADH), cytochrome P450, and aldehyde dehydrogenase (ALDH). Acetaldehyde, a toxic byproduct of alcohol metabolism, damages hepatocytes, activates inflammatory pathways, and disrupts cellular structures, including mitochondria, proteins, and lipids. This cascade can lead to alcoholic steatosis (fatty liver), steatohepatitis, and eventually fibrosis and cirrhosis. Progressive scar tissue formation in cirrhosis disrupts liver architecture and function [9-12].

This study makes a significant contribution to understanding the clinical characteristics and outcomes of men with decompensated alcoholic liver cirrhosis. The results provide a clear picture of the hematological and biochemical abnormalities observed in patients with this disease. Elevated levels of liver enzymes, bilirubin, and D-dimer, along with a high prevalence of anemia and thrombocytopenia, indicate the severity of the condition and its complications. These findings are consistent with previous studies and confirm that alcoholic liver cirrhosis represents a serious public health issue requiring careful diagnosis and treatment [13-20, 20-25].

One of the significant strengths of this study is its extensive and methodologically rigorous design, with large sample size and longitudinal follow-up through outpatient control exams, which allows for tracking disease progression in real-world conditions. Additionally, the study’s setting in a specialized hospital with a gastroenterology and hepatology department ensures precise data collection under controlled conditions. This approach enables a deeper understanding of clinical outcomes, such as variceal bleeding and hepatic encephalopathy, which were identified as major risk factors for mortality in patients with decompensated alcoholic liver cirrhosis. The results of this study support findings from other studies that have identified these complications as key factors in the prognosis and survival of cirrhotic patients [21-29].

Furthermore, it is important to highlight that the large sample size allowed for reliable statistical analysis, which contributes to the validity of the findings. Compared to similar studies, our sample of 123 patients with clearly defined inclusion criteria offers greater precision in the analysis of hematological and biochemical parameters, which may aid in the further personalization of therapeutic approaches for patients with alcoholic liver cirrhosis.

The article "Significance of Laboratory Findings and Esophageal Varices in Male Patients With Decompensated Alcoholic Liver Cirrhosis: A Single-Center Experience" was published in 2025. Journal: Cureus.

It is also crucial to emphasize that the study provides insight into the high mortality rate within the first year of hospitalization, with a particular focus on variceal bleeding as the primary cause of death, which is in line with findings from other studies, including Gu et al. [30], that have identified variceal hemorrhage as a significant risk factor for mortality in cirrhotic patients. These results highlight the importance of preventive measures, such as early identification of varices and appropriate treatment (e.g., beta-blockers), which can significantly reduce the risk of mortality [31,32].

The limitations of this study include its retrospective-prospective design, which may introduce potential selection bias, as well as the exclusion of female patients and those with cirrhosis of other etiologies. While these factors may impact the generalizability of the results, they do not detract from the value of the study, as the focus was on patients with alcoholic liver cirrhosis, a significant subgroup of cirrhosis patients. Additionally, the longitudinal follow-up through outpatient control exams provides a better assessment of long-term outcomes, which is a major strength of this study.

## Conclusions

Our findings provide valuable insights for clinicians treating patients with decompensated alcoholic liver cirrhosis, emphasizing the need for early recognition of complications such as variceal bleeding and intensive monitoring and appropriate treatment. Although there are some limitations, the study lays the foundation for further research into improving patient outcomes through targeted interventions.
